# Aqueous Ginger (*Zingiber officinale*) Extract Ameliorates the Harmful Effects of High-Dose Lornoxicam in Albino Male Rats

**DOI:** 10.1155/2022/1546734

**Published:** 2022-08-02

**Authors:** Sabry M. El-Bahr, Rabab R. Elzoghby, Mohammed A. Alfattah, Mahmoud Kandeel, Ahlam F. Hamouda

**Affiliations:** ^1^Department of Biomedical Sciences, College of Veterinary Medicine, King Faisal University, Al-Ahsa 31982, Saudi Arabia; ^2^Department of Biochemistry, Faculty of Veterinary Medicine, Alexandria University, Alexandria 21523, Egypt; ^3^Department of Pharmacology, Faculty of Veterinary Medicine, New Valley University, Egypt; ^4^Camel Research Center, King Faisal University, Al-Ahsa 31982, Saudi Arabia; ^5^Department of Pharmacology, Faculty of Veterinary Medicine, Kafr Elsheikh University, Egypt; ^6^Department of Forensic Medicine and Toxicology, Teaching Hospital, Faculty of Veterinary Medicine, Benha University, Benha 13736, Egypt

## Abstract

Lornoxicam is a potent oxicam-class nonsteroidal anti-inflammatory drug (NSAID) with analgesic, anti-inflammatory, and antipyretic effects. Its impacts on many biological functions are not fully understood. We measured various biomarkers in male albino rats provided an oral aqueous ginger extract before IM administration of therapeutic and 2× the therapeutic doses of lornoxicam. The aqueous ginger plant extract was characterized by mass spectroscopy, and its effects were determined by examining free radical scavenging activity, blood parameters, renal and hepatic function, semen quality, proinflammatory cytokines, antioxidant markers, and histopathology. Rats administered lornoxicam had significantly higher liver and kidney function biomarker values, TNF-*α*, interleukin-6, and sperm abnormalities than the control rats. The overall erythrocyte count, packed cell volume, prostaglandin, and sperm counts were all considerably lower in the experimental animals. Histological changes were found in the liver, spleen, and testes of rats administered lornoxicam alone. In rats, pretreatment with ginger extract reduced the majority of the negative effects of conventional and high dosages of lornoxicam.

## 1. Introduction

Prevention and treatment of musculoskeletal illnesses are public health priorities in humans and other animals [1]. To treat musculoskeletal injuries, a large variety of anti-inflammatory medications from various chemical classes are commonly used [1], including nonsteroidal anti-inflammatory drugs (NSAIDs), which demonstrate anti-inflammatory and analgesic properties [2]. NSAIDs, including aspirin, ibuprofen, naproxen, and indomethacin, function by suppressing prostaglandin formation [3]. Unfortunately, NSAIDs are also well known to induce liver damage, annually affecting 3 to 23 patients per 100,000 [4]. Because of the identified hepatotoxic side effects, three specific NSAIDs—bromfenac, ibufenac, and benoxaprofen—were removed from the UK and/or US markets [5]. These NSAID-related side effects have been observed in children [6] and older adults [7].

The NSAID lornoxicam (chlorotenoxicam) is an oxicam derivative, suppressing polymorphonuclear (PMN) leukocyte motility, PMN leukocyte superoxide release, and macrophage nitric oxide release [8]. Used in both oral and parenteral forms [9], lornoxicam demonstrates many anti-inflammatory, analgesic [10], and antipyretic properties via the inhibition of two isoforms of the cyclooxygenase enzyme (COX-1 and COX-2) and suppression of prostaglandin (PG) and thromboxane [11]. It also promotes suppression of endotoxin-induced IL-6 production in THP1 monocytes and lower TNF-*α* and IL-1*β* activity.

There are many variables that might lead to an increased risk of NSAID hepatotoxicity, including excessive intake, prescription overdose, drug interactions, and unique patient susceptibilities. [12]. In part to discover natural alternatives to toxic synthetic medications, researchers have investigated the potential of many plants and their extracts to treat various diseases [13]. For example, the active components in many herbs have been revealed as antioxidants that demonstrate low toxicity and high efficacy. One of these herbs is ginger (*Zingiber officinale*).

Medicinal herbs have been utilized to heal various infections since antiquity. According to the World Health Organization, 80 percent of the world's population uses diverse plant fractions and their dynamic ingredients as traditional remedies [14, 15]. The rhizomes of the ginger plant are the most medicinally significant part of the plant [16]. It bears antiarthritic, antiplatelet, antitumor, antioxidant, anti-inflammatory, antiviral, and antihepatotoxic properties [17, 18]. Ginger has been identified as protective against many toxic agents, such as cisplatin [19] and bromobenzene [20], attributed to its ability to increase antioxidant enzyme activity [21]. Researchers discovered a drop in plasma uric acid concentrations after giving ginger extract to broilers [22, 23]. Moreover, rats treated with 2% or 4% dietary ginger for one month demonstrated lower gentamycin-induced nephrotoxicity and renal oxidative stress [24–26]. Ginger ethanolic extracts given in single doses or for several days also protected the animals against nephrotoxicity induced by doxorubicin [27] and cisplatin [19], hepatotoxicity induced by acetaminophen [28] and bromobenzene [20], and testicular toxicity induced by cisplatin [29]. The primary antioxidants in ginger have been identified as 6-gingerol and 6-shogaol [30–32].

The effectiveness of ginger extracts in mitigating the harmful effects of lornoxicam administration has yet to be demonstrated. In addition, the effects of high dosages of lornoxicam (two times the therapeutic dose) on biochemistry, hematological, histology, oxidative stress, cytokine production, and sperm characteristics remain unknown. Therefore, we aimed to investigate the effect of an aqueous ginger extract on these parameters in male albino rats treated with therapeutic and 2× the therapeutic doses of lornoxicam.

## 2. Materials and Methods

### 2.1. Drug and Plant Aqueous Extract

Lornoxicam (16 mg, trade name: Xefo®; 6-chloro-4-hydroxy-2-methyl-N-2-pyridyl-2 H-thieno (2,3-e)-1,2-thiazine-3-carboxamide-1,1-dioxide) was obtained from Eva Pharma Pharmaceuticals Inc. (Cairo, Egypt) in powder form. The powder was diluted in 2 mL of distilled water before to injection, giving a final dosage of 8 mg/mL lornoxicam. Botanists from the Faculty of Agriculture, Benha University, obtained ginger rhizomes from a local market. The rhizomes were crushed in a blender and air-dried. A total of 125 g of air-dried powder was macerated in 200 mL of distilled water for 12 hours at room temperature before filtration to obtain a final aqueous extract concentration of 120 mg/mL for use in the experiment.

### 2.2. Gas Chromatography-Mass Spectrometry (GC–MS) Analysis of the Aqueous Ginger Extract

In the current study, the chemical composition of the aqueous ginger extract was determined using a Trace GC–TSQ mass spectrometer with a direct TG − 5MS 30 m × 0.25 mm × 0.25 *μ*m (film thickness) capillary column (Thermo Scientific, Austin, TX, USA). The components were determined by comparing their relative mass spectra fractions to those of the WILEY 09 and NIST 14 mass spectral databases [33].

### 2.3. DPPH Free Radical Scavenging Activity

The radical-scavenging ability of aqueous ginger extract was evaluated using 2,2-diphenyl-1-picrylhydrazyl (DPPH) as a reagent according to previous studies [34]. To generate DPPH radicals, an ethanol solution of DPPH (1 mM) was generated shortly before the experiment, and 3.9 mL of the DPPH radical solution was mixed in triplicate with 100 L of aqueous ginger extract or 100 L of ethanol (control). The mixture was incubated for 30 min in darkness, and the absorbance was measured spectrophotometrically at 517 nm. Decreased sample absorbance indicates the capacity of the ginger extract to extract DPPH free radicals. The percentage scavenging activity was calculated as percentage inhibition of DPPH (antioxidant capacity% = [absorbance of control–absorbance of sample/absorbance of control] × 100%).

### 2.4. Experimental Animals

Fifty male Wister rats (6–8 weeks old, 225–250 g body weight) were housed in separate cages. The laboratory environment was conventional (temperature 25°C, relative humidity 65%), with a 12-hour light/dark cycle. Throughout the experiment, rats were fed a typical diet of bread, barley and milk, and water ad libitum. For adaption and to prevent stress during the experimental period, the rats were acclimatized to the laboratory conditions for two weeks prior to treatment. The Institutional Animal Care and Use Committee for Research Ethics of Benha University (# BUFVTM3921) approved all study procedures, which followed the principles of the Declaration of Helsinki.

### 2.5. Experimental Design

The 50 rats were divided into five groups of 10 rats. The rats in the first group were given no therapy and served as a control. The rats in the second group were administered IM lornoxicam at a therapeutic dose (0.07 mg/kg/day; [35]) once a day for 10 days. The third group of rats received an oral aqueous extract of ginger (600 mg/kg/day at a concentration of 120 mg/mL; [17, 36]) two hours prior to receiving a therapeutic dose of IM lornoxicam once daily for ten days. The fourth group of rats received a daily IM injection of 2× the therapeutic dose of lornoxicam (0.14 mg/kg/day) for 10 days. The rats in the fifth group were given an aqueous ginger extract (600 mg/kg/day; 120 mg/mL; [17, 36] two hours before receiving an IM injection of double the therapeutic dose of lornoxicam once daily for 10 days.

### 2.6. Hematological Examination

After the end of the experiment, hematological assays were performed on whole blood samples taken from the retroorbital venous plexus. Total erythrocyte count (TEC), packed cell volume % (PCV%), hemoglobin concentration (Hb), mean corpuscular hemoglobin (MCH), mean corpuscular volume (MCV), and mean corpuscular hemoglobin concentration (MCHC) were detected using an automated cell counter (VetScan HM5 Hematology system, Abaxis, Inc., Union City, CA, USA).

### 2.7. Biochemical Examination

Serum samples were used to estimate the activity of alanine aminotransferase (ALT), aspartate aminotransferase (AST), alkaline phosphatase (ALP) [37], catalase (CAT) [38] and glutathione peroxidase (GPX) [39], concentrations of creatinine, [40], urea [41], uric acid [42], and malondialdehyde (MDA) [43]. TNF-*α* and IL-6 concentrations were determined by a commercial ELISA kit [44].

### 2.8. Histopathological Examination

Liver, kidney, testes, and spleen tissue samples were taken from each group's slaughtered animals and processed for histopathological procedures that were performed using standard techniques [45]. Masson's trichrome staining was performed according to a standard protocol [46]. In addition, the epididymis heads were used to measure sperm count [47] and sperm abnormalities [48].

### 2.9. Statistical Analysis

Data were statistically analyzed by one-way ANOVA with a post hoc Duncan multiple comparison test using a statistical software program (SPSS for Windows version 20, IBM, Armonk, NY, USA). Differences were considered significant at a *P* value ≤0.05.

## 3. Results

### 3.1. Characterization of the Aqueous Ginger Extract

GC–MS analysis of aqueous ginger extract indicated that this extract contained nine components: *α*-curcumene, *α*-zingiberene, *β*-sesquiphellandrene, *β*-bisabolene, zingiberene, shogaol, *α*-sitosterol, 6-gingerol, and 2,6,10-dodecatrien-1-ol, 3,7,11-trimethyl (Figure 1). In the DPPH assay, the aqueous ginger extract's antioxidant capacity was 42.79% ± 3.1%.

### 3.2. Liver and Kidney Function Tests

Treatment with lornoxicam at both the therapeutic (group 2) and 2× therapeutic doses (group 4) resulted in significantly higher levels (*P* ≤ 0.05) of kidney function parameters (uric acid, creatinine, and urea; Table 1) and liver function parameters (AST, ALT, and ALP; Table 2) than the nontreated control group. Sera from rats given two times the therapeutic dose of lornoxicam had higher average estimated parameters than those from animals given the therapeutic dose. The increased blood liver and kidney functioning indicators were dramatically improved after treatment with aqueous ginger extract. The amelioration of lornoxicam pathology was observed in all treatment groups, in the following order: group 4 > group 5 > group 2 > group 3.

### 3.3. Hematological Parameters

Therapeutic lornoxicam treatment did not significantly alter the estimated hematological parameters (Table 3). However, rats receiving 2× lornoxicam (group 4) showed significantly reduced RBC count, Hb%, PCV, and WBC count. These changes were significantly improved by treatment with the aqueous ginger extract.

### 3.4. Semen Analysis

Compared with the nontreated control group, treatment with lornoxicam at both the therapeutic and 2× the therapeutic dose (groups 2 and 4, respectively) resulted in significantly lower sperm counts (*P* ≤ 0.05; Table 4), higher % sperm abnormalities, and lower PG levels. Pretreatment with aqueous ginger extract resulted in significantly higher sperm count, lower % sperm abnormalities, and higher PG levels.

### 3.5. Proinflammatory Cytokines and Antioxidant Markers

Compared with the nontreated control group, treatment with lornoxicam at both the therapeutic and 2× the therapeutic doses (groups 2 and 4, respectively) resulted in significantly elevated TNF-*α* and IL-6 levels (*P* ≤ 0.05; Table 5). Pretreatment with aqueous ginger extract significantly decreased TNF-*α* and IL-6 levels. Lornoxicam injection induced a significant reduction of CAT and GPX enzyme activity and increased levels of MDA (Table 5) in the sera of rats of all experimental groups compared to the control (group 1).

### 3.6. Histological Examination

Tables 6–9 showed the effects of ginger (*Zingiber officinale*) aqueous extract on the pathological grading of lornoxicam in renal, hepatic, splenic, and testicular tissues of different treated groups.

#### 3.6.1. Kidney

Histological examination of kidney tissues by H&E staining revealed that control rats (Figure 2(a)) showed less blood vessel congestion than lornoxicam-treated rats (Figure 2(b)). Kidney architecture was restored to normal in rats treated with ginger extract two hours before injection of the therapeutic dose of lornoxicam (Figure 2(c)) and was more intact than that of rats treated with lornoxicam alone (Figure 2(b)). Severe congestion was observed in the kidney tissues of rats treated with the 2× lornoxicam dose alone (Figure 2(d)) compared to the control group (Figure 2(a)). Hydropic degeneration was observed in the kidney tissues of rats pretreated with ginger extract two hours before injection of the 2× lornoxicam dose (Figure 2(e)) compared to control (Figure 2(a)). However, the kidney architecture was more intact than that of rats treated with the 2× lornoxicam dose alone (Figure 2(d)).

#### 3.6.2. Liver

H&E staining of the liver tissues revealed that, unlike the control (Figure 3(a)), lornoxicam alone resulted in a congested central vein (Figure 3(b)). The hepatic structure was normal in rats treated with ginger extract two hours before injection of the therapeutic dose of lornoxicam (Figure 3(c)) and was better than that of rats treated with lornoxicam alone (Figure 3(b)). Hepatic vascular degeneration, sinusoidal dilatation, picnotic and hyperchromatic cells, focal necrosis, mononuclear cellular infiltration, Von Kupffer cell hyperplasia, edema, ballooning, congested hepatic veins, and degenerative changes were observed in the hepatic tissues of rats treated with a 2× lornoxicam dose alone (Figure 3(d)). Only hepatic vein congestion was observed in the liver tissues of rats pretreated with ginger extract before injection of the 2× lornoxicam dose (Figure 3(e)). However, the liver architecture was more intact than in rats treated with 2× lornoxicam dose alone (Figure 3(d)). Results of the PAS reaction were positive in nelson capsules.

#### 3.6.3. Spleen

Compared to the control group (Figure 4(a)), hemorrhage was observed by H&E staining in the splenic tissues of rats injected with a therapeutic dose of lornoxicam alone (Figure 4(b)). The splenic architecture was nearly normal in rats pretreated with ginger extract before receiving the therapeutic dose of lornoxicam (Figure 4(c)) and was more intact than that of rats treated with lornoxicam alone (Figure 4(b)). Hemorrhages with trabecular thickening and hemosiderosis were observed in the splenic tissues of rats treated with a 2× lornoxicam dose alone (Figure 4(d)). Hepatic vein hemosiderosis was observed in splenic tissues of rats pretreated with ginger extract before injection of the 2× lornoxicam dose (Figure 4(e)). However, the splenic architecture was more intact than in rats treated with a 2× lornoxicam dose alone (Figure 4(d)).

#### 3.6.4. Testis

H&E staining of the testicular tissues revealed that, compared to the control (Figure 5(a)), administration of either the therapeutic or 2× lornoxicam dose alone resulted in desquamation in the spermatogonial cells and interstitial edema (Figures 5(b) and 5(d)). Furthermore, apoptosis was detected by Masson's trichrome staining in the testicular tissues of rats injected with either the therapeutic or 2× lornoxicam dose alone (Figures 5(b) and 5(d)) compared to control (Figure 5(a)). In rats given ginger extract two hours before receiving the therapeutic dose of lornoxicam, normal testicular architecture was seen (Figure 5(c)), and the architecture was more intact than in rats treated with lornoxicam alone (Figure 5(b)). Regeneration changes, including the disappearance of interstitial edema and intact spermatogenic cells, were detected in the testicular tissues of rats pretreated with ginger extract before injection of the 2× lornoxicam dose (Figure 5(e)), and the testicular architecture was more intact than in rats treated with a 2× lornoxicam dose alone (Figure 5(d)). A minced epididymis head solution stained with eosin and nigrosin revealed normal sperm heads and tails (Figure 6(a)) in the control group. The following sperm abnormalities were detected in rats administered lornoxicam: abnormal sperm head and tail structure (Figure 6(b)), abnormal sperm head and tail (Figure 6(c)), amorphous head (Figure 6(d)), abnormal head (Figure 6(e)), double head (Figure 6(f)), coiled tail (Figure 6(g)), and double tail (Figure 6(h)).

## 4. Discussion

In the current study, the antioxidant capacity (42.79% ± 3.1%) of the aqueous ginger extract was higher than that detected in a similar, previous study [49] in which the authors observed a DPPH scavenging activity of 16.2%. The highest antioxidant activity percentages detected previously were 79.83%, 70.43%, and 61.70%, observed in red ginger, emprit ginger, and elephant ginger, respectively [50].

Urea is a waste product of protein catabolism produced in the liver and discharged by the kidneys [51], which remove urea and creatinine from the blood through glomerular ultrafiltration, measured by determining the glomerular filtration rate (GFR). Increased urea and creatinine levels in the blood occur from any abnormalities that diminish GFR [52]. We discovered that rats given conventional and high dosages of lornoxicam had higher uric acid levels in their blood than control rats, indicating that lornoxicam had a uricosuric impact. Previous studies similarly reported [53, 54] the uricosuric effect of the NSAID piroxicam, attributed by the authors to increased excretion of uric acid in the urine. The observed increase of serum creatinine after lornoxicam injection was similar to that observed after administration of meloxicam [51] and diclofenac sodium [55, 56] in rabbits. The authors examining the effects of diclofenac sodium proposed that the nephrotoxic effect of this drug was caused by inhibition of cyclooxygenases and subsequent suppression of PG production. Urea, uric acid, and creatinine are general renal biomarkers, and their increased levels indicate kidney injury [55, 56]. Our histopathological results in renal tissues supported the results of our biochemical analyses of kidney function. The improvement of kidney function parameters (uric acid, urea, and creatinine serum concentrations) in rats pretreated with ginger extract two hours before injection of lornoxicam in therapeutic and 2× the therapeutic doses indicates that ginger ameliorated lornoxicam's uricosuric effects [22]. Previously, it is reported that ginger extract reduced uric acid in the plasma of broilers [23]. Furthermore, 2% or 4% of dietary ginger ameliorated nephrotoxic and oxidative stress in rats [24–26]. In the current investigation, the ameliorative effect of ginger was observed in renal tissue histology. Except for hydropic degeneration in the proximal convoluted tubules, the tissue from pretreated rats displayed a more intact morphology. After lornoxicam administration without ginger, we found hydropic degeneration and desquamation of renal epithelial tubules in rat kidney tissues, particularly in rats injected with 2× the therapeutic dose. A previous study [35] similarly demonstrated renal vacuolization and decreased brush borders in proximal tubule epithelia of rats administered lornoxicam. NSAIDs were also found to induce renal vasoconstriction and decrease renal perfusion and acute renal abnormalities due to inhibition of PG biosynthesis [57].

The liver is the major target organ for drug metabolism. Hepatic biotransformation reactions induce hepatocyte apoptosis [58–60]. Therefore, AST, ALT, and ALP activities are commonly used as biomarkers of structural and functional alterations in the liver, which cause levels of these enzymes to increase in the blood [56]. As these enzymes are intracellular, their normal blood concentrations are very low. As a result, hepatocellular damage or necrosis induces an elevation in their blood serum levels [61]. Significant elevations in blood AST, ALT, and ALP were seen in rats injected with lornoxicam alone or in combination with ginger, indicating that the lornoxicam-treated groups had liver abnormalities. The role of ginger extract in improving the liver function enzymes AST, ALT, and ALP of rats injected with lornoxicam was reported previously [62].

In Swiss albino mice, hepatotoxicity, hepatitis, and elevated levels of the liver enzymes AST, ALT, and ALP had previously been documented [63] and rats [64] treated with diclofenac sodium. In addition, there is a high concentration of meloxicam (1 mg/kg/day for five days) and variable (sometimes extensive) necrosis with mild lymphocytic infiltration in rat liver and kidney tissues [65]. Our findings are similarly consistent with the previous research on meloxicam-induced liver injury in animals [66]. Furthermore, the histopathological picture (results of H&E, MTS, and PAS staining) of liver tissues supports the biochemical liver function results. The positive PAS reaction with mucopolysaccharide around the central vein of the liver tissues in nelson capsules indicated inflammation. Marked hepatic dysfunction (fibrotic, necrotic, and apoptotic hepatocytes) was also observed in a previous study of albino rats injected with lornoxicam [67]. Cytochrome P450 isozymes (CYP2C9, CYP2D6, and CYP3A4) metabolize lornoxicam to one of its major metabolites, 5′-hydroxy-lornoxicam, in the liver. This metabolite is responsible for lipid peroxidation and free radical production [68, 69]. This process will consume the GSH available for free radical scavenging. We propose that the consumption of GSH was responsible for the hepatic dysfunction observed in rats in the current study [67].

The protective effect of ginger has been attributed to its relatively high concentration of either vitamin C (35–38 mg per 100 g) [70] or shogaol [71, 72], which participate in antioxidant and antihepatotoxic activities. We identified nine ginger extract components that may contribute to ginger's antioxidant action. In a prior investigation, ginger aqueous extract was found to be protective against adriamycin-induced hepatotoxicity and cisplatin-induced hepatotoxicity [73]. We found that administering ginger extract two hours before lornoxicam injection prevented many alterations in liver architecture in rats (the exception being hepatic vein congestion).

The significant changes in hematological parameters (TEC, Hb, and PCV %) observed in rats treated with lornoxicam at 2× the therapeutic dose may provide evidence of the drug's toxicity. The reduction of red blood cells with subsequent anemia was dose-dependent. This anemia results in reduced oxygen-carrying capacity in the blood and the amount of oxygen delivered to the tissues [74, 75]. Similar significant alterations of hematological parameters were observed in rats treated with diclofenac sodium [75] and paracetamol [74]. Moreover, the induction of anemia may be attributed to the loss of erythrocytes resulting from gastrointestinal bleeding and ulcers [74, 75].

H&E staining of the spleen showed hemorrhage with trabecular thickening and hemosiderosis in splenic tissue of rats injected with 2× the therapeutic dose of lornoxicam without ginger pretreatment. Similarly, N-acetyl-p-aminophenol (140 mg/kg) was found to induce overall splenic congestion, congested sinusoids, widened red pulp, and atrophy of lymphoid follicles [76]. Rats pretreated with ginger had nearly normal blood levels after injection with double the therapeutic dose of lornoxicam. This may be related to high gingerol and shogaol content in the ginger extract [71, 72, 77]. Gingerol has been found to have cardiotonic, analgesic, anti-inflammatory, and antipyretic effects [77], and shogaol acts as an antioxidant [71, 72].

A significant fall in PG levels in rats injected with lornoxicam without ginger pretreatment was previously recorded [78]. Lornoxicam was reported to be 100-fold more potent than tenoxicam in inhibiting PGD2 formation in rat polymorphonuclear leukocytes in vitro [78]. NSAIDs exert anti-inflammatory, antipyretic, and analgesic effects by suppressing PG and thromboxane synthesis [11] via COX enzyme inhibition [24]. In the current study, rats pretreated with ginger extract demonstrated improved prostaglandin levels after injection with lornoxicam, and this may be attributable to the antioxidant effect of ginger's free radical scavenging activity [79, 80].

Previously, it was discovered that aspirin causes hypercholesterolemia in rats via blocking PG production. This inhibition could result in altered cholesterol metabolism and androgen biosynthesis [81]. Androgens are essential for the survival and motility of spermatozoa in the epididymis [82]. In addition, PGs play substantial roles in regulating reproductive activity in males and females [82] and regulate sperm metabolism and function [83]. Aspirin may disrupt spermatogenic processes in the seminiferous tubules, epididymal function, or testosterone's effect on hypothalamic release factors and anterior pituitary gonadotropin production, potentially changing spermatogenesis [84]. In the current study, lornoxicam might have functioned similarly to aspirin [83] and induced morphological abnormalities in sperm cells, but additional studies are required to confirm this mechanism. The considerable decrease in sperm count in rats injected with lornoxicam without ginger pretreatment could be ascribed to cholesterol buildup in the testes. This buildup alters cholesterol metabolism, which impairs sperm dynamics, including spermatogenesis. Similarly, indomethacin was previously proposed to cross blood testis barriers and cause degeneration of seminiferous tubules, focal necrosis, and reduced spermatogenesis [85]. Additional studies are required to determine whether lornoxicam is similar to indomethacin in this regard.

In the current study, lornoxicam injection induced more sperm abnormalities and significantly fewer total sperm than the control. These findings are also reflected in testis histopathology. Desquamation in the spermatogonia and interstitial edema and apoptosis of some cells were the main features identified in rats injected with lornoxicam. A previous study [86] reported similar results in rats injected with indomethacin. We found that ginger extract pretreatment improved the sperm count and decreased sperm abnormalities induced by lornoxicam injection in rats. The regeneration changes exhibited in the testis of rats treated with ginger extract two hours before lornoxicam injection may be attributed to ginger's antioxidant components (gingerol and shogaols) [71, 72, 77].

IL-6 and TNF-*α* are proinflammatory cytokines produced by activated macrophages. They help regulate various biological processes, including cell proliferation, differentiation, apoptosis, immune response, and activation of cell signaling proteins involved in systemic inflammation. The overproduction of TNF-*α* has been implicated in various diseases [87, 88]. Cytokine production may be affected by NSAID interaction with transcriptional factors. In addition, selective COX-2 inhibitors may cause an increase in TNF-*α* levels, probably by inhibiting prostaglandin production [89]. TNF-*α* and IL-6 are widely known to induce hepatorenal toxicity and tissue damage. In previous studies, intoxication with the NSAID paracetamol was found to induce oxidative stress, triggering a secondary inflammatory cascade associated with cytokine release from Kupffer cells [90–92]. Moreover, lornoxicam administration (1.3 mg/kg) in albino rats [93] and acetaminophen in mice [94] were previously associated with significantly increased MDA and cytokines IL-6 and TNF-*α* and significantly decreased CAT and GPX. Furthermore, hepatic GSH, antioxidant enzymes, and lipid peroxidation increased after lornoxicam injection in rats [67]. We propose that the protective effects observed in rats treated with ginger extract two hours before lornoxicam injection resulted from significant reductions of MDA and cytokines (IL-6 and TNF-*α*) and significant elevation of CAT and GPX. This observation may be attributed to the effect of the antioxidant components, gingerol and shogaols, of ginger extract [71, 72, 77, 95, 96]. In a previous study, rats pretreated with ginger (100 mg/kg/day for 14 days) experienced suppressed indomethacin-induced gastric ulceration (single dose, 20 mg/kg, IP). Ginger therapy improved biochemical and histological changes caused by indomethacin, most likely due to increased antioxidant defenses (GSH and SOD) and decreased lipid peroxidation (MDA) [97]. The key protective characteristic of ginger's natural compounds is their suppression of toxin-induced cytokine production (TNF-*α*, IL-6, IL-8, IL-2 and IL-1*β*, PLA2, iNOS, COX-2, and PGE2) [98]. High levels of polyphenolic and flavonoid compounds in ginger extracts might be responsible for the antioxidant and ameliorative activities [99, 100].

## 5. Conclusion

Administration of the therapeutic dose and 2× the therapeutic dose of the NSAID lornoxicam to rats without ginger extract pretreatment resulted in significant increases in the serum activities of ALT, AST, and ALP, concentrations of urea, creatinine, TNF-*α*, and IL-6, and sperm abnormalities. However, RBC, PCV, prostaglandin, and sperm counts were significantly decreased in rats administered lornoxicam without ginger extract pretreatment. Congestion, hydropic degeneration, desquamation, and focal necrosis were observed in the kidney, liver, spleen, and testes of rats administered either lornoxicam dose. All observed detrimental effects were more pronounced in rats receiving 2× the therapeutic dose than those administered the therapeutic dose of lornoxicam. These detrimental effects in rats administered 2× the therapeutic dose of lornoxicam were improved significantly by pretreatment with ginger. We recommend providing a ginger extract pretreatment in animals to avoid any possible hepatic, renal, splenic, and testicular injuries induced by administering a high dose of lornoxicam.

## Figures and Tables

**Figure 1:** The standard curve and components of ginger aqueous extract detected by gas chromatography mass spectrometry analysis.

**Figure 2:** Histological examination of kidney tissues by H&E staining. (a) control (group 1) showed normal renal structure. (b) Group 2 showed congestion in blood vessels. (c) Group 3 showed nearly normal renal architecture. (d) Group 4 showed congestion with hydropic degeneration and desquamation of epithelial renal tubules. (e) Group 5 showed renal tissue return to normal structure except proximal convoluted tubules showed hydropic degeneration (h).

**Figure 3:** Histological examination of liver tissues by H&E staining: (a) control (group 1) showed normal hepatic structure; (b) group 2 showed congested central vein (co); (c) group 3 showed nearly normal hepatic cell architecture; (d) group 4 showed hepatic vascular degeneration, sinusoidal dilatation, picnotic and hyperchromatic cells, focal necrosis sites and mononuclear cellular infiltration, Von Kupffer cell hyperplasia, necrotic, apoptotic of hepatocelluar appearance, edema and ballooning degenerative changes (de), and congested hepatic veins; and (e) group 5 showed the hepatic architecture restored to normal except hepatic veins congestion (co). Positive PAS reaction (arrow).

**Figure 4:** Histological examination of spleen tissues by H&E staining: (a) control (group 1) showed normal spleen structure, (b) group 2 showed hemorrhage (co), (c) group 3 showed nearly normal spleen architecture, (d) group 4 showed hemorrhage with trabecular thickening with hemosiderosis (t), and (e) group 5 showed the hepatic architecture restored to normal except decreased number of hemosiderosis (h).

**Figure 5:** Histological examination of testicular tissues by H&E staining: (a) control (group 1) showed normal testes structure, (b) group 2 showed normal structure except desquamation in the spermatogonile cells and interstitial edema of some cells and sings of apoptosis (Masson technique; o), (c) group 3 showed nearly normal testicular architecture, (d) group 4 showed desquamation in the spermatogonile and interstitial edema and sings of apoptosis (Masson technique; o), and (e) group 5 showed regeneration changes include disappearance of interstitial edema and the spermatogenic cells returned to be intacted to the basement membrane.

**Figure 6:** Microscopic examination of head of epididymis minced solution in rats stained with Eosin & Nigrosin stain: (a) normal sperm head and tail and (b) abnormal sperm head and tail, (c) abnormal sperm head and tail, (d) amorphous head, (e) abnormal head, (f) double head, (g) coiled tail, and (h) double tail.

**Table 1:** Effects of ginger (*Zingiber officinale*) aqueous extract on kidney function of lornoxicam treated male albino rats.

Groups	Uric acid (mg/dl)	Creatinine (mg/dl)	Urea (mg/dl)
1	3.13 ± 0.01^e^	0.69 ± 0.02^e^	20.89 ± 1.50^e^
2	6.70 ± 0.03^c^	1.15 ± 0.02^c^	47.09 ± 1.16^c^
3	5.99 ± 0.04^d^	0.99 ± 0.02^d^	44.25 ± 0.96^d^
4	8.79 ± 0.03^a^	2.01 ± 0.07^a^	55.35 ± 1.69^a^
5	7.44 ± 0.06^b^	1.37 ± 0.03^b^	50.18 ± 1.36^b^

^a-e^The values represented as mean ± SD. Means within the same column followed by different letters are significantly different (*P* ≤ 0.05).

**Table 2:** Effects of ginger (*Zingiber officinale*) aqueous extract on liver function of lornoxicam treated male albino rats.

Groups	AST, U/mL	ALT, U/mL	ALP, U/mL
1	26.09 ± 1.60^e^	104.31 ± 2.53^e^	151.33 ± 5.58^e^
2	44.42 ± 1.6^c^	293.72 ± 2.72^c^	228.67 ± 3.49^c^
3	40.47 ± 1.5^d^	273.0 ± 2.47^d^	221.33 ± 2.62^d^
4	57.71 ± 1.35^a^	511.62 ± 5.08^a^	404.67 ± 4.13^a^
5	48.34 ± 1.87^b^	397.04 ± 9.25^b^	343.67 ± 3.84^b^

The values represent mean ± SD. Means within the same column followed by different letters are significantly different (*P* ≤ 0.05).

**Table 3:** Effects of ginger (*Zingiber officinale*) aqueous extract on hematological indices of lornoxicam treated male albino rats.

Groups	RBC×106/*μ*L	HB gm/dl	PCV%	WBC×103 *μ*L
1	7.69 ± 0.29^a^	13.86 ± 2.79^a^	38.57 ± 1.28^a^	12.13 ± 3.2^a^
2	7.02 ± 0.25^a^	11.43 ± 1.47^a^	35.89 ± 1.47^a^	10.8 ± 2.82^a^
3	7.66 ± 0.62^a^	12.03 ± 1.97^a^	36.20 ± 1.93^a^	11.10 ± 1.15^a^
4	3.10 ± 0.21^b^	7.50 ± 0.58^b^	25.67 ± 1.74^b^	3.50 ± 1.10^b^
5	6.82 ± 1.28^a^	10.17 ± 1.23^a^	31.72 ± 2.36^a^	10.58 ± 2.16^a^

The values represent mean ± SD. Means within the same column followed by different letters are significantly different (*P* ≤ 0.05).

**Table 4:** Effects of ginger (*Zingiber officinale*) aqueous extract on semen analysis and Prostaglandins concentration of lornoxicam treated male albino rats.

Groups	Sperm, million/gm	Sperm abnormalities %	Prostaglandins, ng/mL
1	6.23 ± 0.35^a^	8.67 ± 0.88^e^	2360.21 ± 4.89^a^
2	4.18 ± 0.10^c^	13.33 ± 0.45^c^	948.90 ± 3.46^c^
3	5.37 ± 0.07^b^	11.33 ± 0.20^d^	1017.3 ± 5.46^b^
4	3.35 ± 0.07^e^	25.10 ± 0.31^a^	663.57 ± 7.64^e^
5	4.50 ± 0.06^d^	18.50 ± 0.32^b^	891.67 ± 6.01^d^

The values represent mean ± SD. Means within the same column followed by different letters are significantly different (*P* ≤ 0.05).

**Table 5:** Effects of ginger (*Zingiber officinale*) aqueous extract on oxidative stress and cytokines of lornoxicam treated male albino rats.

Groups	MDA, nmol/gm	CAT, U/gm	GPX, U/gm	TNF-*α*, pg/mL	IL6, pg/mL
1	137.55 ± 5.3^e^	628.29 ± 7.4^a^	588.84 ± 4.5^a^	43.84 ± 1.79^e^	26.37 ± 0.33^e^
2	182.61 ± 3.5^c^	521.19 ± 5.2^c^	422.14 ± 4.6^c^	98.58 ± 1.58^c^	33.97 ± 1.71^c^
3	173.79 ± 2.8^d^	534.32 ± 6.1^b^	534.88 ± 5.1^b^	88.93 ± 2.42^d^	30.16 ± 0.68^d^
4	283.98 ± 2.8^a^	498.54 ± 3.4^e^	369.08 ± 3.8^e^	147.85 ± 5.67^a^	49.60 ± 2.28^a^
5	253.04 ± 2.6^b^	502.69 ± 4.9^d^	401.93 ± 5.4^d^	123.19 ± 7.15^b^	37.51 ± 1.27^b^

The values represent mean ± SD. Means within the same column followed by different letters are significantly different (*P* ≤ 0.05).

**Table 6:** Effects of ginger (*Zingiber officinale*) aqueous extract on the pathological grading of lornoxicam in renal tissue of different treated groups.

Groups	Number	Pathological grading			
		0	I	II	III
1	10	10	0	0	0
2	10	0	4	4	2
3	10	5	1	2	2
4	10	0	2	4	4
5	10	5	1	2	2

**Table 7:** Effects of ginger (*Zingiber officinale*) aqueous extract on the pathological grading of lornoxicam in hepatic tissue of different treated groups.

Groups	Number	Pathological grading			
		0	I	II	III
1	10	10	0	0	0
2	10	0	3	3	4
3	10	4	2	3	1
4	10	0	2	4	4
5	10	5	1	3	1

**Table 8:** Effects of ginger (*Zingiber officinale*) aqueous extract on the pathological grading of lornoxicam in splenic tissue of different treated groups.

Groups	Number	Pathological grading			
		0	I	II	III
1	10	10	0	0	0
2	10	0	5	4	1
3	10	5	2	2	1
4	10	0	2	4	4
5	10	5	3	1	1

**Table 9:** Effects of ginger (*Zingiber officinale*) aqueous extract on the pathological grading of lornoxicam in testicular tissue of different treated groups.

Groups	Number	Pathological grading			
		0	I	II	III
1	10	10	0	0	0
2	10	0	4	4	2
3	10	5	1	2	2
4	10	0	2	4	4
5	10	5	1	2	2

## Data Availability

All data generated or analyzed during this study are included in this article.
